# Effect of Coronavirus Disease (COVID-19) on Human Semen: No Evidence of Coronavirus in Semen of Patients

**DOI:** 10.1155/2022/6204880

**Published:** 2022-09-12

**Authors:** Serajoddin Vahidi, Ali Nabi, Hojat Alipoor, Hormoz Karami, Amirhossein Rahavian, Alireza Ayatollahi, Laleh Dehghan Marvast, Saeid Abouei

**Affiliations:** ^1^Andrology Research Center, Yazd Reproductive Science Institute, Shahid Sadoughi University of Medical Sciences, Yazd, Iran; ^2^Department of Urology, Shahid Sadoughi University of Medical Sciences, Iran; ^3^Department of Urology, Shahid Sadoughi University of YAZD, Iran

## Abstract

**Background:**

In December 2019, a severe acute respiratory syndrome (SARS-COV-2) was found in China. The coronavirus can impact different organs, as shown by the virus having been detected in urine, blood, oropharyngeal, and feces. This study was done to assess the impact of COVID-19 on semen analysis and to evaluate the existence of the virus in the semen of infected men. *Methodology*. Forty fertile men with COVID-19 were confirmed by an oropharyngeal sample. The men were divided into two groups. The semen of twenty men in the acute stage of COVID-19 and twenty men in the clinical recovery stage was analyzed, and the parameters of semen were compared between two groups. In addition, a PCR test of patients' semen was done.

**Result:**

The analysis showed that all patients' semen specimens tested negative. Semen analysis revealed no significant difference in sperm count, concentration, or motility, and the sperm of both groups was found to be normal. However, viability and morphology parameters were significantly lower in men with the acute disease.

**Conclusion:**

Coronavirus (COVID-19) was not secreted in the semen of infected men but had a negative effect on the morphology and viability of the sperm of men in the acute stage.

## 1. Introduction

In December 2019, an outbreak of unexplained pneumonia in Wuhan China was caused by a new coronavirus infection named coronavirus disease 2019 (COVID-2019) [1, 2]. Patients had clinical symptoms, including cough and fever [3]. Research on the new coronavirus was initially focused on quick and accurate identification of the virus, and eventually, real-time reverse-transcriptase polymerase chain reaction (rRT-PCR) was chosen as the gold standard for diagnosis [1]. The virus has been detected in urine, blood, oropharyngeal, and feces (digestive system) [4]. The study of COVID-19 quickly became one of the most important tasks of humanity because of its vastly negative effect on many different organs, including lung, liver, thyroid, spleen, heart, renal, and testis, and its high rate of transmission [4, 5]. Only a few studies have evaluated the impact of the coronavirus on the genital system, and these results have been inconclusive, with some articles mentioning a positive sample test for COVID-19 in the semen of men [6] and other studies reporting negative results [7, 8]. A few types of research have compared the impact of COVID-19 on semen parameters of men in the acute and clinical recovery stage of the infection [9]. This study was designed to detect the virus in semen of infected men during the acute and clinical recovery stage and also to evaluate the impact of this infection on sperm parameters of patients during these two disease stages.

## 2. Materials and Methods

This study was performed on men with COVID-19 infection confirmed by an rRT-PCR from an oropharyngeal sample [10]. We recruited 70 fertile men who have had COVID-19 from August 2021 to December 2021 and have had children within the last two years. The participants were made up of 40 men in the acute disease stage but not hospitalized and 30 men in the clinical recovery stage who had not been hospitalized in their acute stage period. The men had completed the acute period of their illness at least 1 month to a maximum of 3 months. Patients with testicular damage, testicular infection, and testicular surgery and those who were above the age of 45 or under 18 were excluded. In total, 20 men in the acute stage and 20 men in the clinical recovery stage were accepted for this study.

All candidates were trained so they could provide an accurate sample. The sample room was sterilized before each use, and all the candidates were required to wear a mask and wash and dry their hands and penis completely. All the samples were first placed in an incubator (Heracell 150i) in the laboratory. Then, lipofection was mixed with a viral transport medium (VTM) ((gen azma pajouhan Isatis (GAPA), Yazd, Iran)). Lastly, a PCR test was performed on all the sample to detect the virus in the semen fluid. Semen analysis (WHO 2010 protocol) was performed by one person. The treated and control groups were statistically compared using the Kolmogorov-Smirnov test, independent *t*-test, and Mann-Whitney test. All analyses were performed in SPSS version 16, with a *P* value < 0.05 considered significant. Written consent was obtained from each patient. This study was performed and approved by the Medical Ethical Committee of the Research Center for Infertility-Shahid Sadoughi University of Medical Sciences (IR.SSU.RSI.REC.1400.010).

## 3. Result

After applying inclusion and exclusion criteria, we identified that 20 out of the 40 patients were in the acute stage; the rest were in clinical recovery. While all the patients tested positive for SARS-COV-2-RNA in oropharyngeal swab specimens, they all tested negative in semen specimens. While the mean age of the patients in the acute group was found to be higher, it was not significantly higher (35.05 ± 0.21 vs. 33.9 ± 6.82, *P* value: 0.98). The BMI, smoking history, and past medical history of the two groups were not found to be significantly different.

Tables 1 and 2 show the results of the semen analysis. As can be seen, there was no significant difference in the sperm count or other motility parameters between the acute and clinical recovery groups. However, a significant difference in the viability and morphology parameters can be observed. According to the WHO 2010 protocol, the viability and morphology of the participants in clinical recovery were normal despite there was not reported in the acute stage.

## 4. Discussion

Previous studies have shown that severe respiratory syndrome coronavirus (SARS-COV-2), the causal agent of the disease called coronavirus 2019 (COVID-19), can involve multiple organ systems, including the respiratory system, digestive system, and hematological system [11]. COVID-19 has been detected in urine, anal, and oropharyngeal swabs [4].

In this study, we investigated the existence of coronavirus in human semen and compared the impact of the illness on semen analysis between acute and clinical recovery groups. The results of this study did not detect SARS-COV-2 in the semen of adult Iranian males in either the acute or clinical recovery groups, and because of this result, there is no chance of transfer during sex. In contrast, another study reported SARS-COV-2 in the semen of men [6]. In that study, 6 of the 38 recruited patients tested positive for SARS-COV-2. On closer inspection, it was found that the patients in that study had been hospitalized, and the positive samples may have been contaminated during collection. There is also a hypothesis that states testicular injury and inflammatory infiltration viral orchitis can lead to the secretion of COVID-19 in semen [9, 6]. Our results are similar to Song et al. [9], Omolaoye et al. [12], Pan et al. [8], and Fraietta et al. [13] with negative findings for COV-2 in semen samples. Conversely, Li et al. reported positive sample COV-2 status in some patients [6].

Some studies reported a significant difference in semen analysis between the two groups (acute and clinical recovery group); these studies explain their divergent results as a limitation of age and the exclusion of varicocele and hospitalized patients in the acute stage. One of the main goals of this study was to attempt to find and compare the impact of COVID-19 on semen analysis between patients in the acute and clinical recovery stages. The semen analyses showed no significant difference between the two groups in semen count or motility parameters; however, the analyses revealed significant differences between the two groups in viability and morphology parameters. The morphology and viability in the clinical recovery group were better (see Tables 1 and 2), in contrast to the results of previous studies showing abnormal semen analyses parameters in patients who had been infected with coronavirus (COVID-19) [9, 14]. Ma et al.'s study described semen characteristics and mentioned 33.3% (4/12 patients) had lower sperm motility than normal, but they did not have a control or comparing group [15]. Holtmann et al. compared the semen analysis of patients with mild and moderate infections (needing hospitalization, two groups after recovery, and a control group that never got SARS-COV-2). They reported statistically significant impairment of sperm quality between the men recovered from a moderate infection, men who recovered from a mild infection, and the control group [14].

One possible reason the semen analysis was impaired in the acute stage and not in the clinical recovery stage could be stress. This disease, like many other acute diseases, greatly impacts the body, which can cause a temporary disorder in spermatogenesis, and after passing through this acute stage, the situation will return to its normal state [16].

We also showed morphology and viability were impaired in the acute stage. This needs to be estimated and followed up in patients after the acute stage to be confirmed by a second semen analyses in the clinical recovery stage.

This study is limited by the lack of previous semen analyses from the recruited men. And to counter this limitation and in order to compare the conditions between the two groups, we recruited men who have had children within the last two years in lieu of a previous normal semen analysis.

## 5. Conclusion

In summary, we confirm the lack of SARS-COV-2 in the semen of males in the acute and clinical recovery stage. Nevertheless, our findings would seem to show differences in some viability and morphology parameters between the acute and clinical recovery status; also, the study needs to be done with a larger group of participants to confirm the results are generalizable.

## Figures and Tables

**Table 1:** Parameters in sperm analysis.

Variable	Group	Mean	STD deviation	*P* value
Count	1	69.25	37.09	0.983
	2	69.00	34.91	

Progressive	1	45.65	12.25	0.098
	2	38.35	14.81	

Immotile	1	44.15	12.34	0.070
	2	52.05	14.36	

Viability	1	69.55	11.54	0.041
	2	41.60	12.73	

1: clinical recovery group; 2: acute group; *P* values < 0.05 are significant.

**Table 2:** Morphology and nonprogressive in semen analysis.

Variable	Group	Median	Interquartile range	*P* value
Nonprogressive	1	9.00	3	0.826
	2	9.00	3	

Morphology	1	5.00	5	0.021
	2	3.00	1	

1: clinical recovery group; 2: acute group; *P* values < 0.05 are significant. The parameters of the table did not have normal distribution.

## Data Availability

We confirm that all of the material methods and data are available.
